This article has been retracted.

# Effect of Tegretol on Oxidative Stress, Serum Inflammatory Factors, and Left Ventricular Function in AMI Patients after Emergency PCI

**DOI:** 10.1155/2022/8929058

**Published:** 2022-08-02

**Authors:** Liping Ma, Yizhan Pan, Ziying Wu, Lin Zhang, Zhaojin Feng, Ketao Li

**Affiliations:** Shulan (Hangzhou) Hospital Affiliated to Zhejiang Shuren University, Shulan International Medical College, #848 Dongxin Road, Hangzhou, China 310000

## Abstract

To investigate the effects of tegretol on oxidative stress, serum inflammatory factors, and left ventricular function in patients with acute myocardial infarction (AMI) after emergency percutaneous coronary intervention (PCI), 70 AMI patients who received PCI in the emergency department of our hospital from January 2021 to December 2021 were collected. The patients in the control group were treated with aspirin, clopidogrel, and heparin sodium during the perioperative period, and the patients in the study group were treated with tegretol. The levels of oxidative stress, serum inflammatory factors, and left ventricular function index were compared between the two groups. The patients in the control group were treated with TT ((12.00 ± 2.05) s), APTT ((35.50 ± 4.19) s), PT ((16.60 ± 1.58) s), TT ((15.90 ± 2.14) s) APTT ((30.40 ± 3.80) s), and PT ((14.30 ± 1.45) s)) and were comparable (*P* > 0.05), and the difference was statistically significant (*t* = 8.210, 4.600, 7.010, *P* < 0.001). There was no comparable difference in the level of oxidative stress index before treatment (*P* > 0.05). After treatment, there was significant difference in MDA ((14.53 ± 2.14) mmol/L), SOD ((120.45 ± 8.17) U/L), MDA ((11.15 ± 2.02) mmol/L), and SOD ((129.86 ± 8.55) U/L) in the control group (*t* = 7.320, 5.099, *P* < 0.001). The levels of inflammatory factors in patients before treatment were not comparable (*P* > 0.05). After treatment, there were levels of IL-6 ((3.20 ± 1.05) ng/L), CRP ((4.80 ± 1.16) mg/L), MPO ((196.78 ± 21.51) mg/L) and TNF-*α* ((3.96 ± 0.80) pmol/L), IL-6 ((1.95 ± 0.80) ng/L), CRP ((3.10 ± 1.02) mg/L), MPO ((163.60 ± 21.10) mg/L), and TNF-*α* in a study group level ((3.05 ± 0.70) pmol/L), with statistically significant difference (*t* = 5.187, 6.028, 6.031, 4.689,*P* < 0.001). Before treatment, there was no comparable difference in the level of left ventricular function index (*P* > 0.05). After treatment, there was significant difference in LVEF ((46.10 ± 2.39) %) and LVDD ((52.06 ± 1.07) mm), LVEF ((56.85 ± 2.33) %), and LVDD ((48.75 ± 1.02) mm) in the control group (*t* = 17.640, 21.540, *P* < 0.001). Tegretol as an adjunctive therapy for emergency PCI patients with acute myocardial infarction can effectively improve postoperative coagulation function, reduce oxidative stress and inflammatory reaction, and improve cardiac function indicators. It has a positive clinical value.

## 1. Introduction

In clinical practice, AMI is a frequent myocardial necrosis disease whose physiopathological basis is mostly myocardial blood flow disruption, coronary atherosclerosis, and platelet aggregation, which is accompanied by severe chest pain and a high mortality rate [1]. The current clinical treatment for AMI in China mainly uses PCI, which can successfully restore myocardial blood perfusion and minimize myocardial ischemia and ischemia/hypoxia-induced loss [2]. However, due to the effects of platelet aggregation and activation and damage to vascular endothelial cells by PCI in AMI patients, postoperative thrombosis is highly likely to form and cause a second heart attack [3]. Studies have shown that the occurrence and development of AMI are closely related to inflammatory factors and oxidative stress [4, 5].

The use of antiplatelet agents before emergency PCI in patients with AMI can effectively inhibit platelet activity which may reduce the rate of postoperative complications [6]. Tegretol is a novel antiplatelet aggregation drug that exerts antiplatelet effects without catalytic enzyme biotransformation which is outstanding in improving coronary blood flow velocity and reducing myocardial injury [7, 8].

At present, there are few reports on the changes of serum inflammatory factor level, oxidative stress index, and right ventricular function index in patients with AMI before and after treatment with tegretol. Given this, the present adjuvant therapy of tegretol in our patients with AMI who had undergone emergency PCI achieved satisfactory results, and the drug use is reported as follows.

## 2. Materials and Methods

### 2.1. General Information

Seventy AMI patients treated with PCI in our hospital in the emergency department between January 2021 and December 2021 were divided into two groups (each *n* = 35) by the random number table: 19 males and 16 females in the control group, aged 40-69 years, mean age (of 53.10 ± 1.40) years, while 20 males and 15 females in the study group, aged 40-70 years, with mean age (the data differences were comparable (*P* > 0.05)), and this study was approved by the hospital ethics committee.

### 2.2. Inclusion and Exclusion Criteria

#### 2.2.1. Inclusion Criteria

(1) Patients met the criteria for AMI diagnosis [9], and the time between admission and treatment did not exceed 6 h. (2) All patients were first-time patients, and patients voluntarily enrolled after learning about the study.

#### 2.2.2. Exclusion Criteria

The exclusion criteria were as follows: (1) viral myocarditis, heart valve disease, heparin dysfunction, malignancy, and systemic infectious diseases; (2) mental illness that can lead to ineffective communication with the patient and allergic to drugs used in this study or related contraindications; (3) this includes bleeding constitutional or contraindications to bleeding, entrapment aneurysm, severe hypotension, severe trauma, or history of surgery within 2 weeks; and (4) poor compliance, withdrawal, or death in the middle of the study.

### 2.3. Methods

In the control group, there were aspirin (manufacturer: Shenyang Original Pharmacolabo Co., Ltd., NMPN: H20065051, specification: 100 mg^∗^24 s), clopidogrel (manufacturer: Lepu Pharmaceuticals, Inc. Co., Ltd., NMPN: H20123116, specification: 25 mg^∗^10 s^∗^2 plates), and heparin sodium (manufacturer: Sanofi (Beijing) Pharmaceutical Co., Ltd., State Drug Administration: J20180035, specification: 2 sticks (0.4 ml: 4000 AxalU)) for adjuvant therapy. Patients were instructed to take aspirin (300 mg) and clopidogrel (150 mg) orally before surgery; heparin sodium (100 U/kg) was administered intravenously during surgery; clopidogrel was administered twice daily for 7 d after surgery, 75 mg each time, and aspirin was administered once daily, 100 mg each time.

The study group was treated perioperatively with tegretol (manufacturer: Nanjing Zhengda Tianqing Pharmaceutical Co., Ltd., NMPN: H20193177, specification: 90 mg^∗^14 tablets) as adjuvant therapy. Preoperative aspirin was used in the same way as the control group, tegretol (180 mg); intraoperative intravenous push use of heparin sodium was used in the same way as the control group; postoperative tegretol was used twice a day for 7 d, 90 mg each time, and aspirin was used in the same way as the control group.

### 2.4. Observation Indexes

Before and after treatment, 3 ml of fasting venous blood was collected from patients by nurses in the early morning, and the changes in TT, APTT, and PT were tested with the aid of a fully automated hemagglutination device.

Before and after treatment, nurses drew 3 ml of fasting venous blood from patients in the early morning, centrifuged, and processed for MDA levels using the thiobarbituric acid (TBA) method and SOD levels using the enzyme rate method.

Before and after treatment, the nurses tested the patients' IL-6, CRP, MPO, and TNF-*α* levels using the enzyme-linked immunosorbent assay (ELISA).

Pre- and posttreatment tests were performed to compare patients' LVEF and LVDD.

### 2.5. Statistical Analysis

SPSS statistics (version 20.0) was used for data analysis. The measurement data were expressed in (*x* ± *s*). The blood coagulation index, oxidative stress index, inflammatory factor, and left ventricular function index between the two groups were compared by Student's *t*-test. The statistical significance level was determined as *P* < 0.05.

## 3. Results

### 3.1. Comparison of Coagulation Index Levels in Patients

The differences in coagulation index levels of patients before treatment were comparable (*P* > 0.05), and after treatment, TT levels in the study group were lower than those in the control group, and APTT and PT levels were higher than those in the control group, with statistically significant differences (*P* < 0.001), see Table 1.

### 3.2. Comparison of Oxidative Stress Index Levels in Patients

The differences in oxidative stress index levels of patients before treatment were comparable (*P* > 0.05), and after treatment, the MDA levels of the study group were lower than those of the control group, and the SOD levels were higher than those of the control group, with statistically significant differences (*P* < 0.001), as shown in Table 2.

### 3.3. Comparison of Inflammatory Factor Levels in Patients

The differences in inflammatory factor levels of patients before treatment were comparable (*P* > 0.05), and after treatment, the levels of inflammatory factors in the study group were lower than those in the control group, and the differences were statistically significant (*P* < 0.001), as shown in Table 3.

### 3.4. Comparison of Patients' Left Ventricular Function Index Levels

The differences in the levels of left ventricular function indexes of patients before treatment were comparable (*P* > 0.05), and after treatment, the LVEF of the study group was higher than that of the control group, and the LVDD was lower than that of the control group, with statistically significant differences (*P* < 0.001), as shown in Table 4.

## 4. Discussion

Currently, PCI is the therapy of choice for patients with AMI in domestic emergency clinics, since it may successfully relieve myocardial ischemia symptoms and minimize myocardial damage while unblocking coronary arteries [10]. Platelet activity aggregation has been demonstrated to play a crucial role in the development and progression of AMI, according to research [11]. After emergency PCI in AMI patients, the patient's platelet level remains in a state of continuous activation, and a considerable number of aggregates adhere to the coronary stent, which is especially sensitive to postoperative coronary stent thrombosis (ST), resulting in no postoperative reflow, which may adversely influence myocardial blood flow microcirculation reperfusion and surgical outcomes [12]. Therefore, antiplatelet agents should be used to reduce platelet activity aggregation before emergency PCI for AMI. Clopidogrel is a regularly used antiplatelet medicine with considerable benefits in clinical practice; although, it is difficult to work quickly since it must be catalyzed by enzymes in the body before exerting its pharmacological effects. Recently, clinical use of tegretol has been introduced, which is a new type of antiplatelet drug, and the antiplatelet effect can be exerted in a short period after entering the body, thus making it more suitable for emergency treatment of AMI [13].

During emergency PCI for AMI patients, the stenting process and the ballooning process will cause damage to the endothelial cells, and the atherosclerotic material will be released after the exposure of intimal collagen, which will stimulate thrombin and lead to a large number of platelet adhesions and aggregation, which will affect the coagulation function of the body, making the disease more difficult to treat and affect the prognosis, which will lead to in-stent restenosis in serious cases, since AMI patients themselves have poor coagulation function. APTT, TT, and PT are often used clinically to assess coagulation function. Related studies have shown that coagulation is in a low expression state after emergency PCI treatment in patients with AMI. Antiplatelet therapy is therefore particularly critical. Tegretol is a representative third-generation thrombolytic drug, which can improve specific thrombolysis with the help of gene and protein technology, and is particularly suitable for the treatment of AMI because of its fast thrombolysis and dredging speed, high thrombolytic efficiency, and long drug half-life time [14]. This study showed that the differences in coagulation index levels of patients before treatment were comparable (*P* > 0.05), and after treatment, TT levels in the study group were lower than those in the control group, and APTT and PT levels were higher than those in the control group, with statistically significant differences (*P* < 0.001). The results suggest that adjuvant therapy of tegretol in patients with AMI after emergency PCI is excellent in improving coagulation function in patients.

Clopidogrel is a frequently used antiplatelet aggregation drug in clinical practice. However, the drug requires activation of cytochrome P540 enzyme before it can bind to platelet P2Y12, and hepatic metabolism has a large impact on its efficacy, making its efficacy variable and prone to resistance. Tegretol is a precursor drug, and the mechanism of action of the drug is similar to that of clopidogrel, since tegretol itself is the active form, and does not require hepatic metabolism, the onset of action of the drug is significantly earlier than clopidogrel, the use of 2 h can weaken the platelet activity, and metabolic enzyme genetic polymorphism does not affect it; there is no drug resistance, and it has a strong antiplatelet effect, especially suitable for clopidogrel low-response patients. Compared with clopidogrel, the former can reversibly inhibit P2Y12 without causing permanent platelet inactivation, and platelet function can be gradually restored after drug discontinuation; so, the improvement of postoperative coagulation function is more satisfactory, and the inhibition of P2Y12 can be reduced. In addition, P2Y12 receptors are mainly distributed on the surface of inflammatory cells, and tegretol can facilitate the antiplatelet pathway to enhance the anti-inflammatory effect on the organization of free radical production, thus being able to effectively reduce postoperative oxidative stress damage [15]. This study showed that the differences in the levels of oxidative stress indexes in patients before treatment were comparable (*P* > 0.05), and after treatment, the MDA levels in the study group were lower than those in the control group and the SOD levels were higher than those in the control group, with statistically significant differences (*P* < 0.001). The results suggest that adjuvant therapy of tegretol in patients who had undergone emergency PCI for AMI is effective in improving the levels of oxidative stress indexes in patients.

Adenosine is an endogenous anti-inflammatory substance with an inhibitory effect on IL-6 formation and the ability to act directly at the granulocyte surface A2a receptor to provide relief from oxygen radical release. A related study [16] showed that adenosine has an ameliorating effect on postischemic myocardial contractile function in rats which can block inflammatory factors such as TNF-*α* due to cardiomyocyte-mediated postischemia reperfusion. Tegretol increases plasma adenosine levels, indirectly increasing coronary blood flow and improving vascular endothelial function while decreasing the inflammatory response. The study showed that the differences in inflammatory factor levels of patients before treatment were comparable (*P* > 0.05), and after treatment, the levels of inflammatory factors in the study group were lower than those in the control group, with statistically significant differences (*P* < 0.001). In patients having emergency PCI for AMI, the data indicate that adjuvant tegretol treatment is effective in decreasing inflammatory factor levels and improving the inflammatory response.

Aspirin and clopidogrel are often used clinically to combat platelet aggregation. Aspirin can inhibit the conversion of arachidonic acid into thromboxane A2 to play an antidrug role, while clopidogrel can inhibit the binding of adenosine diphosphate to platelet receptors to block the platelet activation pathway, and these two drugs are often used together to achieve the purpose of dual antiplatelet therapy (DAPT). Tegretol is effective within 30 min of oral use, whereas clopidogrel takes 2 h to take effect orally, making tegretol more suitable for perioperative use in AMI patients who had undergone emergency PCI. The long-term efficacy of tegretol is significa clopidogrel than that of clopidogrel since it can promote improved cardiac function and reduce the occurrence of major adverse cardiovascular events (MACE) in patients. Related studies [17] concluded that clopidogrel has less effect on platelet levels, with rapid drug onset, ideal effect in improving cardiac function, and more promising application. This study showed that the differences in the levels of left ventricular function indexes of patients before treatment were comparable (*P* > 0.05), and after treatment, the LVEF of the study group was higher than that of the control group, and the LVDD was lower than that of the control group, with statistically significant differences (*P* < 0.001). The results suggest that adjuvant therapy of tegretol in patients who had undergone emergency PCI for AMI does not unduly affect platelet levels and facilitates improvement in cardiac function.

In conclusion, the use of tegretol adjuvant therapy in patients who had undergone AMI emergency PCI can effectively improve patients' postoperative coagulation function, reduce oxidative stress and inflammatory response, and promote the improvement of cardiac function; therefore, this pharmacotherapy has a positive promotion value in clinical practice.

## Figures and Tables

**Table 1:** Levels of coagulation indexes in comparison patients (*S*, *x* ± *s*).

Groups	Number of cases	TT		APTT		PT	
		Before treatment	After treatment	Before treatment	After treatment	Before treatment	After treatment
Control group	35	6.35 ± 1.11	12.00 ± 2.05	25.80 ± 3.15	34.50 ± 4.19	11.29 ± 1.25	16.60 ± 1.58
Study group	35	6.36 ± 1.13	15.90 ± 2.14	25.78 ± 3.13	30.40 ± 3.80	11.30 ± 1.22	14.30 ± 1.45
*t*	/	0.155	8.210	0.060	4.600	0.101	7.010
*P*	/	0.874	<0.001	0.955	<0.001	0.910	<0.001

**Table 2:** Levels of sclerotic stress indexes in comparison patients (*x* ± *s*).

Groups	Number of cases	MDA level (mmol/L)		SOD level (U/L)	
		Before treatment	After treatment	Before treatment	After treatment
Control group	35	20.54 ± 3.20	14.53 ± 2.14	89.60 ± 6.12	120.45 ± 8.17
Study group	35	20.55 ± 3.18	11.15 ± 2.02	89.92 ± 6.10	129.86 ± 8.55
*t*	/	0.170	7.320	0.410	5.099
*P*	/	0.855	<0.001	0.685	<0.001

**Table 3:** Levels of inflammatory factors in comparison patients (*x* ± *s*).

Groups	Number of cases	IL-6 levels (ng/L)		CRP level (mg/L)		MPO level (mg/L)		TNF-*α* level (pmol/L)	
		Before treatment	After treatment	Before treatment	After treatment	Before treatment	After treatment	Before treatment	After treatment
Control group	35	4.70 ± 1.20	3.20 ± 1.05	6.95 ± 0.92	4.80 ± 1.16	242.29 ± 23.89	196.78 ± 21.51	7.65 ± 1.05	3.96 ± 0.80
Study group	35	4.72 ± 1.19	1.95 ± 0.80	6.97 ± 0.90	3.10 ± 1.02	242.27 ± 23.92	163.60 ± 21.10	7.66 ± 1.07	3.05 ± 0.70
*t*	/	0.065	5.187	0.085	6.028	0.003	6.031	0.037	4.689
*P*	/	0.949	<0.001	0.932	<0.001	0.997	<0.001	0.971	<0.001

**Table 4:** Levels of left ventricular function indexes in comparison patients (*x* ± *s*).

Groups	Number of cases	LVEF (%)		LVDD (mm)	
		Before treatment	After treatment	Before treatment	After treatment
Control group	35	42.10 ± 1.12	52.10 ± 2.39	57.18 ± 1.17	52.06 ± 1.07
Study group	35	42.08 ± 1.15	60.85 ± 2.33	57.20 ± 1.15	48.75 ± 1.02
*t*	/	0.068	17.640	0.067	21.540
*P*	/	0.946	<0.001	0.947	<0.001

## Data Availability

The simulation experiment data used to support the findings of this study are available from the corresponding author upon request.
